RETRACTED

# Research on the Difference between Environmental Music Perception and Innovation Ability Based on EEG Data

**DOI:** 10.1155/2022/9441697

**Published:** 2022-11-17

**Authors:** Na Zhang

**Affiliations:** School of Education Science, Shanxi Normal University, Taiyuan 041009, China

## Abstract

It is of great significance to practice and explore music creation for training creative talents. Perception includes feeling and perception, and feeling is a reflection of individual attributes of objective things directly acting on sensory organs. This paper mainly has a research on the difference between environmental music perception and innovation ability based on EEG data. First, this study performed noise reduction and artifact preprocessing of EEG signals generated by subjects with different levels of consciousness subjected to musical stimulation and then performed tensor decomposition to obtain the tensor component of EEG. The time-domain components of these tensor components were analyzed together with five musical features (fluctuation centroid, fluctuation entropy, pulse clarity, key clarity, and mode), EEG tensor components related to music characteristics were analyzed, the power spectrum and the distribution of responsive brain regions were analyzed, and finally, the differences in the processing of music characteristics by different levels of consciousness were explored.

## 1. Introduction

Brain processing of music is a hierarchical neural processing process that extracts the low-level features of sound and then abstracts the high-level musical structure [1]. In recent years, the relationship between music perception and consciousness has become one of the concerns in the field of cognitive science. The exploration of the relationship between music perception and consciousness is helpful to reveal the neural mechanism of human brain cognitive activities, and it is also of great significance to the clinical application of music therapy. Previous studies on music perception are based on the state of consciousness, such as using awake subjects' functional magnetic resonance imaging (fMRI), to study the brain regions activated by music [2] and utilizing event-related potential (ERP) to study the changes in ERP response in waveform and rhythm of music perception [3]. There are also studies on the mental activity of patients with clear consciousness and brain injury when listening to music [4]. With the introduction of the concepts of microconsciousness state (MCS) and vegetative state (VS) as natural models of consciousness disorders, these two states of consciousness provide a new model and research paradigm for exploring the relationship between music perception and consciousness. Previous studies on subjects in different states of consciousness who were subjected to sound stimulation showed that the electroencephalogram (EEG) features [5], mismatch negative waves (MMN) [6], and functional magnetic resonance responses [7] showed differences in cortical responses. In recent years, many novel research methods have emerged, including EEG signal processing methods and music informatics feature analysis methods, which provide a new perspective for exploring the relationship between music perception and consciousness. Cong et al. used tensor decomposition to extract multidimensional features of EEG signals when listening to music and verified the feasibility [8]. EEG signal is a mixture of a large number of neural signals superimposed, so before studying the relationship between musical features and EEG signal, we must first extract the neural activity components related to musical features from EEG. Tensor decomposition is a multidimensional blind source separation method, which decomposes EEG signals into multiple independent source components with multidimensional characteristics, and each independent source component is an independent neural activity [9]. Compared with other blind source separation methods (such as independent component analysis), tensor decomposition can make use of mathematical model algorithm in multidimensional feature space to separate the collected mixed signals into various independent tensor components while retaining multidimensional features of signals, such as time domain, frequency domain, and spatial distribution [10–12]. Finally, by calculating the temporal correlation between components and music features, the neural activity related to music features is screened, and then the EEG components responding to music features are obtained. In addition, acoustic features (intensity, pitch, and timbre) were used to study musical features. In 2012, Alluri et al. proposed the concept of time-domain signal characteristics of music from the perspective of signal based on local melody and range characteristics of music, including fluctuation centroid, fluctuation entropy, pulse clarity, key clarity, and mode [13]. Alluri et al. combined these musical features to study the fMRI of the tested music and found that a large-scale brain activity involving cognitive, motor, and limbic circuits was activated when the brain processed these musical features [13]. This brings the study of music perception from the traditional acoustic paradigm to the level of signaling and provides a new perspective for the paradigm of brain mechanism of music processing. Based on the new technology of EEG signal analysis and the characteristics of music informatics (signal), this study carried out a research on the difference in music perception of different states of consciousness and revealed how the state of consciousness affects the brain's processing of music production. By designing music stimulation experiments, collecting relevant brain telegrams, and using hierarchical alternating least squares (HALS) nonnegative CP tensor decomposition algorithm, dissociate music-related tensor components from collected EEG. Finally, the ratio power spectrum analysis and spatial distribution analysis of each EEG tensor component were performed to understand the influence of different levels of consciousness on brain processing music characteristics.

RETRACTED

## 2. EEG Acquisition Method

### 2.1. Selection of Experiment Subjects

In this study, the EEG signals of the subjects in the microconscious state group and the vegetative state group were collected from Hangzhou Mingzhou Brain Health Rehabilitation Hospital and Hangzhou Hospital of Zhejiang Armed Police Corps. None of the selected subjects needed intubation and ventilator-assisted breathing, and they had no history of cardiopulmonary resuscitation or mental illness. In addition, in order to ensure the stability of the subjects' consciousness state and the consistency of EEG characteristics during the study, subjects who were in the microconsciousness state or vegetative state for more than one month and in the chronic stage were selected [14]. At the same time, the following case characteristics were excluded: patients with moderate or higher hearing loss, patients with locked-in syndrome, and patients with diseases that may lead to neuropathic deficits in the brain. In the evaluation of consciousness level in this study, the CRS-R scale, which is effective in the international classification of microconscious state and vegetative state, was used as the quantitative tool of consciousness level, and 6 items whose scores were less than 4-5-6-3-2-3 were screened out. The subjects were divided into three groups: normal subjects group, microconscious state group, and vegetative state group. The normal group consisted of 7 subjects aged 20–30 years. There were 17 people in the microconscious state group and 19 people in the vegetative state group, and their ages ranged from 20 to 55. The details of the subjects in the microconscious state group and the vegetative state group are shown in Table 1.

### 2.2. Signal Acquisition Scheme

A 64-lead ActiveTwoSystem EEG acquisition instrument produced by BioSemi was used in the experiment, and the sampling rate was 2048 Hz. The data was collected in monopole lead mode, and A1 and A2 were selected as reference electrodes. According to the international 10/20 standard lead system, electrodes were placed on the scalp surface of the subject, and conductive gel was injected between the electrodes and scalp to make the resistance less than 5 K·*ω*.

RETRACTED

After the subjects entered the quiet state, the EEG acquisition experiment began. The EEG signals of the subjects in the resting state were collected for 60 s at first, then 120 s in the state of music stimulation, and finally 60 s in the resting state after stimulation. The stimulation source of this study is the climax chorus of Jasmine Flower, which is 120 s in length and plays at a sound level of 70 dB. In the experiment, the subjects listened to music with their eyes closed. For the subjects with consciousness impairment who could not close their eyes, they covered their eyes with a towel. During the acquisition process, there is no noise and high-power electrical equipment dry disturbance. The subjects were in repose, and the room temperature was controlled at 25°C.

### 2.3. EEG Preprocessing

In this study, EEGLAB Version 13_5_4B was used to analyze EEG signals on Matlab 2019A platform. Firstly, the EEG was filtered by depower frequency. According to the current frequency in China, the depower frequency was set to 50 Hz. Secondly, according to the rhythm characteristics of EEG, the cut-off frequency of bandpass filtering was set as low pass 80 Hz and high pass 0.5 Hz. According to EEGLAB, the waveform after filtering was observed, and the large disturbance and muscle artifact were removed so as to obtain the EEG signal after denoising. After noise reduction, the signal will still have artifacts, such as electrooculogram (EOG). Based on Matlab 2016a, ICASSO toolbox was used as the signal partition solution method based on InfomaxICA, and independent component analysis (ICA) was implemented for the EEG after noise reduction to remove artifacts.

## 3. Extraction of Musical Features

Matlab2016a was used to compile and translate environment, and MIRtoolbox version 1.7.1 was added to extract 5 acoustic and musical characteristics of stimulus source Jasmine Flower. It includes fluctuation centroid, fluctuation entropy, pulse clarity, key clarity, and mode [13, 15]. Firstly, the window shifting method was used to sample music from zero seconds by using the window width of 3 s and overlapping with the front and rear windows of 2 s each [16]. Then, using MIRToolbox, the values of acoustic characteristics (fluctuation centroid, fluctuation entropy, pulse clarity, key clarity, and mode) of each acoustic segment are calculated.

## 4. EEG Feature Extraction

### 4.1. Calculation of Third-Order Tensor of EEG Signal

The spatial distribution (channel), time domain, and frequency domain of EEG signal are selected as the characteristics of the third-order tensor. In order to obtain the time-frequency domain characteristics of each lead of EEG signal of each subject as the third-order component of the tensor, short-time Fourier transform was used for time-frequency domain analysis of the signal [11]. The EEG signals of each lead were sampled by hamming window, which was 3 s wide and overlapped with front and rear windows for 2 s each. Thus, the size of the third-order tensor of each EEG signal is channel × frequency × time, where channel = 64, frequency = 158, and time = 120-artifact time, where artifact time refers to the time of removing part of signal due to large artifact during preprocessing.

RETRACTED

### 4.2. Nonnegative CP Tensor Decomposition Based on HALS

Canonical polyadic (CP) decomposition and Tucker decomposition can be used to extract high-dimensional tensor components of signals. CP decomposition is the process of decomposing a given n-order tensor *X* into the sum of a series of rank tensor quantities. According to the order, tensors can be divided into first-order vectors, second-order matrices, and third-order and higher-order tensors. Similar to matrix decomposition, an n-order tensor *X* can be decomposed into the sum of *R* n-order tensor of rank [17]. Each rank tensor is a component of a tensor. A tensor of rank *N* is equal to the cross product of *N* orthogonal unit vectors times the energy coefficient. Thus, the CP decomposition of a tensor *X* of order *N* can be obtained as follows:

(1) $$\begin{array}{c} X=\sum_{r=1}^{R}\lambda_{r}\cdot \alpha_{r1}\cdot \alpha_{r2}\Lambda \alpha_{rN}, \end{array}$$

where the tensor *X* is a tensor of order *N*, *λ*_*r*_ is the energy coefficient, and *α*_*r*1_, *α*_*r*2_, Λ, *α*_*rN*_ are the orthogonal unit vectors, and the symbol represents the tensor cross product. Nonnegative CP tensor decomposition is used in this study to decompose the third-order tensors obtained in Section 4.1 of this paper. In this process, a series of optimal nonnegative orthogonal vector combinations are approached continuously so that the remaining tensor norm ‖*E*‖^2^ approaches zero. The calculation process of the two norms of the remaining tensor ‖*E*‖^2^ is as follows:

(2) $$\begin{array}{c} {\left\|E\right\|}^{2}={\left\|X-\sum_{r=1}^{R}\lambda_{r}\cdot \alpha_{r1}\cdot \alpha_{r2}\cdot \alpha_{r3},\right\|}_{F}^{2}. \end{array}$$

In order to accelerate the convergence of the remaining tensor binary norm and reduce the dependence of computation force, the hierarchical alternating least squares (HALS) optimization process of nonnegative CP tensor decomposition is selected in this study [18].

RETRACTED

### 4.3. Extraction and Screening of EEG Tensor Components

In Section 4.2 of this paper, the nonnegative CP tensor decomposition algorithm based on HALS is introduced. This algorithm will be used to decompose the third-order signal tensor of each subject obtained in Section 4.1 of this paper to obtain the components of brain electrical activity. The number of tensor components is extracted from the signal tensor and determined by Smooth DIFFIT [19]. All the tensor components extracted by the above methods contain three components, which are spatial distribution coefficient, time-domain envelope, and spectrum. The brain topographic map was drawn according to the spatial distribution coefficient of the tensor components, and then the tensor components satisfying the dipolar form were screened out, namely, the EEG tensor components [10, 20]. Then, the time-domain envelope components of the tensor components were analyzed by Pearson correlation coefficient with the five kinds of music time-domain characteristic values obtained in method 2. The threshold value of the correlation coefficient was calculated by the Monte Carlo method, and the components related to music characteristics were selected (*P* < 0.05). That is, the electrical activity of the brain corresponds to changes in musical characteristics [8, 11, 13].

### 4.4. Ratio Power Spectrum Analysis and Statistical Test

The EEG tensor obtained in Section 4.3 of this paper has three components: spatial distribution coefficient, time-domain envelope, and spectrum, among which the frequency domain component of the EEG tensor reflects the spectral characteristics of the component. According to the frequency domain component, the specific power spectrum, that is, the proportion of each node law, can be calculated to analyze whether the EEG signals of subjects with different levels of consciousness respond to music characteristics in rhythm. The ratio power spectrum of each rhythm is calculated as follows:

(3) $$\begin{array}{c} \text{ratio}=\frac{\int_{f_{2}}^{f_{1}}\text{psd}\left(\tau \right)d_{\tau }}{\int_{1}^{30}\text{psd}\left(\tau \right)d_{\tau }}, \end{array}$$

where F1 and F2 are the lower limit and upper limit of frequency band of interest, respectively, namely, delta (1–4 Hz), theta (4–8 Hz), alpha (8–13 Hz), and beta (13–30 Hz). The spatial distribution component of the EEG tensor component represents the distribution of the component in the brain region. The higher the coefficient is, the closer the sampling point is to the source component that generates the EEG tensor component. Thus, the location of the responsive brain region where the source component occurs can be determined by a brain program. SPSS V.20 (SPSS Inc. Chicago, IL), ANOVA factor assay, and Scheffe's postassay for power spectrum ratios of EEG tensor components; *P* < 0.05 was considered statistically significant. Finally, the differences in the distribution of power spectrum and response brain regions of unrelated and related EEG tensor components were compared, and it was excluded that the differences in power spectrum and brain topography of the three groups were not related to music perception but may be caused by the differences in their own consciousness level.

RETRACTED

## 5. Experimental Results

Through the tensor decomposition algorithm in Section 4 and the tensor component screening method in Section 4.3, 18 components were screened out from 7 normal subjects, 41 components were screened out from 17 cases of microconscious state, and 32 components were screened out from 19 cases of vegetative state. The results are shown in Table 2.

### 5.1. Ratio Power Spectrum Analysis and Statistical Test of EEG Tensor Components Related to Musical Features

According to the method proposed in this paper, all the EEG tensor components related to musical features were analyzed by ratio power spectrum analysis. Tables 3–7 show the ratio power spectrum analysis results of EEG tensor components associated with the fluctuation centroid, fluctuation entropy, pulse clarity, key clarity, and mode musical features, respectively.

Table 3 shows the average power spectrum of EEG tensor component ratio related to music feature fluctuation centroid. The proportions of alpha and beta waves in normal subjects were higher than that of theta and delta waves, while the proportions of theta and delta waves in minimally conscious and vegetative states were higher than that of alpha and beta waves. The proportions of alpha and beta waves of EEG tensor components of the three groups were statistically different (alpha wave: *F* (2, 21) = 104.838, *P* < 0.001; beta wave: *F* (2, 21) = 10.418, *P*=0.001). The alpha wave proportion of the EEG tensor component in the normal group was higher than that in the microconscious state group (*P* < 0.001) and vegetative state group (*P* < 0.001). The beta wave proportion of the EEG tensor component in the normal group was higher than that in the microconscious state group (*P* < 0.001) and vegetative state group (*P* < 0.001). There was no difference in the proportion of EEG tensor components in each rhythm band between the microconscious state group and the vegetative state group.

Table 4 shows the average power spectrum of the EEG tensor component ratio related to music feature fluctuation entropy. Since there are only two EEG tensor components related to fluctuation entropy in the normal group and the vegetative state group, independent sample statistical analysis is not performed. However, it can be observed that the proportion of alpha and beta waves in the normal group is higher than that of theta and delta waves, and the EEG tensor components in the microconscious state group and the vegetative state group are opposite. The alpha wave proportion of EEG tensor in the normal group was higher than that in the microconscious state group and vegetative state group. There was no difference in the proportion of EEG tensor in each rhythm band between the microconscious state group and the vegetative state group.

RETRACTED

Table 5 shows the average power spectrum of EEG tensor component ratios associated with the musical feature key clarity. The proportions of alpha and beta waves in normal subjects were higher than that of theta and delta waves, while the proportions of theta and delta waves in minimally conscious and vegetative states were higher than that of alpha and beta waves. There were statistical differences in the alpha and beta proportions of EEG tensor components among the three groups (alpha wave: *F* (2, 18) = 27.349, *P* < 0.001; beta wave: *F* (2, 18) = 6.758, *P*=0.006). The alpha wave proportion of the EEG tensor component in the normal group was higher than that in the microconscious state group (*P* < 0.001) and vegetative state group (*P* < 0.001). The beta wave proportion of the EEG tensor component in the normal group was higher than that in the microconscious state group (*P*=0.010) and vegetative state group (*P*=0.022). There was no difference in the proportion of EEG tensor in each rhythm band between the microconscious state group and the vegetative state group.

Table 6 shows the average power spectrum of EEG tensor component ratios associated with music feature pulse clarity. The proportions of alpha and beta waves in the normal group were higher than that of theta and delta waves, while the proportions of theta and delta waves in the slightly conscious state group and the vegetative state group were higher than that of alpha and beta waves. There were statistical differences in the alpha and beta wave proportions of EEG tensor components among the three groups (alpha wave: *F* (2, 21) = 27.349, *P* < 0.001; beta wave: *F* (2, 18) = 6.758, *P*=0.006). The alpha wave proportion of the EEG tensor component in the normal group was higher than that in the microconscious state group (*P* < 0.001) and vegetative state group (*P* < 0.001). The beta wave proportion of the EEG tensor component in the normal group was higher than that in the microconscious state group (*P*=0.01) and vegetative state group (*P*=0.022). There was no difference in the proportion of EEG tensor in each rhythm band between the microconscious state group and the vegetative state group.

RETRACTED

Table 7 shows the mean power spectrum of the EEG tensor component ratio related to musical feature mode. The proportions of alpha and beta waves in normal subjects were higher than that of theta and delta waves, while the proportions of theta and delta waves in minimally conscious and vegetative states were higher than that of alpha and beta waves. There was a statistical difference in the proportion of alpha wave of EEG tensor components among the three groups (alpha wave: *F* (2, 6) = 5.79, *P*=0.040). There was no difference in the proportion of EEG tensor components in each rhythm band between the microconscious state group and the vegetative state group.

### 5.2. Statistical Analysis of the Distribution of EEG Tensor Components in Response Brain Regions Related to Music Features

According to the spatial distribution coefficient component of the EEG tensor obtained in this paper, the brain topographic map can be drawn, and the responsive brain regions of the EEG tensor can be determined. Tables 8–10 show the distribution statistics of EEG tensor components related to music characteristics in the normal group, the microconsciousness state group, and the vegetative state group, respectively. In the normal group, the EEG tensors were distributed in the prefrontal lobe except 2 in the temporal lobe. In the microconscious group, only 6 EEG tensors were distributed in the prefrontal lobe, and the rest were mainly located in the temporal lobe. In the vegetative state group, only one EEG tensor was distributed in the prefrontal lobe, and the rest were mainly distributed in the temporal lobe. As shown in Figure 1, from left to right are the brain maps of the normal group with the response brain region of the prefrontal lobe tensor component, the brain maps of the microconscious state group with the response brain region of the temporal lobe tensor component, and the brain maps of the implant state group with the response brain region of the temporal lobe tensor component, respectively.

### 5.3. Statistics and Analysis of Ratio Power Spectrum and Distribution of Response Brain Regions of EEG Tensor Components Unrelated to Music Features

In this section, the ratio power spectrum and response brain area distribution statistics of EEG tensor components unrelated to music characteristics were conducted in the three groups of subjects so as to exclude the possibility that the power spectrum and brain topographic map of the three groups of subjects were only caused by their different levels of consciousness and had nothing to do with music perception. There were 145 EEG tensor components in the normal group, 202 in the microconscious state group, and 307 in the vegetative state group.

RETRACTED

Table 11 shows the mean power spectrum of the ratio of EEG tensor components unrelated to musical features of the three groups of subjects. The proportion of delta waves in the vegetative state group (0.629 ± 0.372) was higher than that in the microconscious state group (0.436 ± 0.385) and the normal control group (0.183 ± 0.265) (*F* (2,640) = 77.179, *P* < 0.001). The proportion of theta wave in the microconscious state group (0.240 ± 0.298) and the vegetative state group (0.213 ± 0.293) was higher than that in the normal control group (0.124 ± 0.157) (*F* (2,640) = 8.494, *P* < 0.001). The proportion of alpha waves in the normal group (0.483 ± 0.320) was higher than that in the microconscious state group (0.081 ± 0.121) and vegetative state group (0.056 ± 0.092) (*F* (2,640) = 308.538, *P* < 0.001). Beta wave proportion in the normal group (0.159 ± 0.105) was higher than that in the microconscious state group (0.025 ± 0.021) and the vegetative state group (0.029 ± 0.036) (*F* (2,640) = 299.129, *P* < 0.001).

Table 12 shows the ratio power spectrum of EEG tensor components unrelated to music characteristics and the distribution of response brain regions in the three groups. In the normal group, 97 of 145 EEG tensor components were located in the prefrontal lobe. In the microconscious group, 44 of the 202 EEG tensor components were located in the prefrontal lobe, and 51 of the 307 EEG tensor components were located in the vegetative state group.

The ratio power spectrum of EEG tensor components unrelated to musical features was compared with the ratio power spectrum of EEG tensor components unrelated to musical features, and the ratio power spectrum of EEG tensor components unrelated to musical features was compared with the ratio power spectrum of EEG tensor components unrelated to musical features in Section 5.2. First of all, there was no difference in the proportion of delta waves of the EEG tensor related to music in the microconscious state group and the vegetative state group, while the proportion of delta waves of the EEG tensor unrelated to music in the microconscious state group was lower than that in the vegetative state group. Second, the theta wave proportion of the EEG tensor related to music in the normal group was lower than that in the microconscious and vegetative state groups, while the theta wave proportion of the EEG tensor unrelated to music in the normal group and the microconscious and vegetative state groups was different. Finally, the microconsciousness and vegetative state groups and music characteristics of unrelated electrical tensor component proportion of response to a brain region located in the frontal lobe are higher than electrical tensor components related to music features, and normal controls associated with the time-domain characteristics of music electrical tensor component proportion of response to a brain region located in the frontal lobe are higher than the time-domain characteristics of the music not related electrical tensor components.

RETRACTED

Therefore, by comparing the EEG tensor components unrelated to the temporal characteristics of music with those related to music, it can be seen that the two components of the response brain region distribution and power spectrum are different in the statistical results of the three groups of subjects. Based on this, according to the experimental results, it is concluded that the differences in power spectrum and brain topography of the three groups of subjects are related to music perception, not only caused by the differences in their own consciousness level.

In this study, the EEG signals generated by the subjects with different levels of consciousness under the stimulation of music were preprocessed with noise reduction and deartifacts. Then, based on the nonnegative CP tensor decomposition of HALS, the processed signals were decomposed by tensor decomposition to obtain the tensor components of the EEG. The time-domain component of the tensor component separately with five kinds of music features (fluctuation centroid, fluctuation entropy pulse clarity key clarity, and mode) and correlation analysis to extract the characteristics of music-related electrical tensor components, the power spectrum, and the distribution of response brain regions were analyzed. Finally, the differences in musical feature processing in different levels of consciousness were explored. According to the power spectrum of EEG tensor components related to music and the distribution of response brain regions in the three groups, it can be seen that there are differences in the rhythm and response brain regions of the subjects under music stimulation. In terms of rhythm, the ratio power spectrum analysis of the components obtained by tensor decomposition showed that, except for characteristic mode, the proportion of alpha wave and beta wave in response to EEG tensor components in normal conscious state was higher than that in the microconscious state and vegetative state. There was no significant difference in the proportion of each rhythm between the microconscious state and the vegetative state. In the normal conscious state, the proportion of alpha and beta waves responding to EEG tensor was higher than that of delta and theta waves, while in the microconscious state and vegetative state, the proportion of delta and theta waves was higher than that of alpha and beta waves. Based on previous studies on EEG rhythm, attention and high-intensity cognitive activity can cause the appearance of beta waves, and the present study found that the beta rhythm of EEG tensor components related to music in the microconscious state and vegetative state was significantly less than that in the normal conscious state. It can be speculated that the two groups of conscious states have weaker perception and attention to musical features. In terms of the response brain regions, the response brain regions in the normal state of consciousness were mainly concentrated in the prefrontal lobe, while the response brain regions in the microstate of consciousness and vegetative state were mainly in the temporal lobe. This means that as the level of consciousness decreases, the response of the prefrontal lobe decreases, while the temporal lobe basically maintains, supporting the importance of the prefrontal lobe for consciousness. For the brain mechanism of music processing, Koelsch proposed a hierarchical music processing model. According to this theory, it can be concluded that the normal state of consciousness to the fourth stage of music structure processing did not happen in a state of consciousness and plants because the fourth stage structure of musically activated processing is located in the prefrontal cortex, neither the conscious state nor the vegetative state is activated by the prefrontal cortex. Secondly, this study compared the frequency domain characteristics of components occurring in the temporal lobe of normal conscious state, microconscious state, and vegetative state and found that the responses of the three groups of subjects to the music characteristics of the EEG tensor components in rhythm distribution were different. The alpha and beta waves of EEG tensor in the normal conscious state were still higher than delta and theta waves, while theta and delta waves were the main components of EEG tensor in the microconscious state and vegetative state. This suggests that the level of consciousness decreases, and so does the temporal lobe's electrical rhythm in response to musical features.

RETRACTED

## 6. Conclusion

It was found that the responses of normal subjects, microconscious subjects, and vegetative subjects to musical features were different in rhythm and response region. In terms of brain activation area distribution, the response of normal subjects to music was mainly concentrated in the prefrontal lobe, while the response of microconscious and vegetative state subjects to music was concentrated in the temporal lobe. In terms of rhythm distribution, the EEG response frequency of normal subjects to musical features was concentrated in alpha and beta bands, while the EEG response frequency of microconscious and vegetative state subjects was concentrated in theta and delta bands.

## Figures and Tables

**Figure 1:** Spatial component of EEG tensor components correlated with musical feature. (a) Normal group; (b) MCS group; (c) VS group.

**Table 1:** Information about MCS and VS participants.

Functional state of brain	Number of people	Age	CRS-R score	Microconscious or vegetative state time/month	Gender
					Men or women
Microconscious state	17	53.82 ± 15.26	12.82 ± 4.14	3.10 ± 1.92	125
Vegetative state	19	47.79 ± 13.26	5.53 ± 2.37	4.05 ± 1.38	145

**Table 2:** Statistics on the number of EEG tensor components correlated with five musical features among different consciousness level groups.

Grouping	Fluctuation centroid	Fluctuation entropy	Key clarity	Pulse clarity	Mode
Normal group	5	2	5	3	3
Microconscious state group	12	9	7	10	3
Plant state group	7	3	9	10	3

**Table 3:** The mean value of the power spectrum ratio of EEG tensor components correlated with the music feature fluctuation centroid.

Grouping	Delta wave	Theta wave	Alpha wave	Beta wave
Normal group	0 039 ± 0 055	0 096 ± 0 091	0 687 ± 0 193	0 170 ± 0 104
Microconscious state group	0.573 ± 0.405	0.279 ± 0.342	0.033 ± 0.022^*∗∗*^	0.027 ± 0.017^*∗∗*^
Plant state group	0.479 ± 0.442	0.390 ± 0.384	0.063 ± 0.040^*∗∗*^	0.053 ± 0.067^*∗∗*^

*Note.* ^*∗*^ *P* < 0.05; ^*∗∗*^*P* < 0.01.

**Table 4:** The mean value of the power spectrum ratio of EEG tensor components correlated with the music feature fluctuation entropy.

Grouping	Delta wave	Theta wave	Alpha wave	Beta wave
Normal group	0 017 ± 0 024	0 046 ± 0 018	0 588 ± 0 132	0 380 ± 0 119
Microconscious state group	0.706 ± 0.307	0.138 ± 0.127	0.041 ± 0.025	0.031 ± 0.024
Plant state group	0.474 ± 0.433	0.387 ± 0.358	0.085 ± 0.077	0.080 ± 0.095

**Table 5:** The mean value of the power spectrum ratio of EEG tensor components correlated with the music feature key clarity.

Grouping	Delta wave	Theta wave	Alpha wave	Beta wave
Normal group	0 038 ± 0 085	0 047 ± 0 056	0 668 ± 0 295	0 115 ± 0 056
Microconscious state group	0.454 ± 0.392	0.152 ± 0.287	0.096 ± 0.103^*∗∗*^	0.032 ± 0.021^*∗*^
Plant state group	0.519 ± 0.414	0.345 ± 0.406	0.057 ± 0.065^*∗∗*^	0.044 ± 0.043^*∗*^

*Note.* ^*∗*^ *P* < 0.05; ^*∗∗*^*P* < 0.01.

**Table 6:** The mean value of the power spectrum ratio of EEG tensor components correlated with the music feature pulse clarity.

Grouping	Delta wave	Theta wave	Alpha wave	Beta wave
Normal group	0 035 ± 0 012	0 054 ± 0 041	0 672 ± 0 064	0 226 ± 0 072
Microconscious state group	0.327 ± 0.412	0.349 ± 0.373	0.144 ± 0.242^*∗∗*^	0.026 ± 0.021^*∗*^
Plant state group	0.561 ± 0.425	0.299 ± 0.361	0.044 ± 0.044^*∗∗*^	0.029 ± 0.024^*∗*^

*Note.* ^*∗*^ *P* < 0.05; ^*∗∗*^*P* < 0.01.

RETRACTED

**Table 7:** The mean value of the power spectrum ratio of EEG tensor components correlated with the music feature mode.

Grouping	Delta wave	Theta wave	Alpha wave	Beta wave
Normal group	0 118 ± 0 054	0 183 ± 0 015	0 432 ± 0 273	0 267 ± 0 218
Microconscious state group	0.414 ± 0.451	0.466 ± 0.429	0.057 ± 0.049^*∗*^	0.014 ± 0.008
Plant state group	0.589 ± 0.522	0.337 ± 0.515	0.033 ± 0.026^*∗*^	0.014 ± 0.012

*Note.* ^*∗*^ *P* < 0.05; ^*∗∗*^*P* < 0.01.

**Table 8:** The number of locations of EEG tensor components correlated with musical feature in the normal group.

	Frontal lobe	Temporal lobe	Parietal lobe	Posterior occipital lobe	Total
Fluctuation centroid	4	1	0	0	5
Fluctuation entropy	1	1	0	0	2
Key clarity	5	0	0	0	5
Pulse clarity	3	0	0	0	3
Mode	3	0	0	0	3
Total	16	2	0	0	18

**Table 9:** The number of locations of EEG tensor components correlated with musical feature in the MCS group.

	Frontal lobe	Temporal lobe	Parietal lobe	Posterior occipital lobe	Total
Fluctuation centroid	1	9	1	1	12
Fluctuation entropy	1	7	0	1	9
Key clarity	1	2	3	1	7
Pulse clarity	2	5	2	1	10
Mode	1	1	0	1	3
Total	6	24	6	5	41

**Table 10:** The number of locations of EEG tensor components correlated with musical feature in the VS group.

	Frontal lobe	Temporal lobe	Parietal lobe	Posterior occipital lobe	Total
Fluctuation centroid	0	5	1	1	7
Fluctuation entropy	0	0	3	0	3
Key clarity	0	5	2	2	9
Pulse clarity	1	6	2	1	10
Mode	0	1	1	1	3
Total	1	17	9	5	32

**Table 11:** The mean value of the power spectrum ratio of EEG tensor components not correlated with the music feature.

	Delta	Theta	Alpha	Beta
Normal group	0.183 ± 0.265	0.124 ± 0.157	0.483 ± 0.320	0.159 ± 0.105
Microconscious state group	0.436 ± 0.385^*∗*##^	0.240 ± 0.298^*∗∗*^	0.081 ± 0.121^*∗∗*^	0.025 ± 0.021^*∗∗*^
Plant state group	0.626 ± 0.373^*∗*##^	0.214 ± 0.293^*∗∗*^	0.056 ± 0.092^*∗∗*^	0.029 ± 0.036^*∗∗*^

*Note. P* < 0.05 versus normal group, ^*∗∗*^*P* < 0.01 versus normal group, and ^*##*^*P* < 0.01 MCS group versus VS group.

**Table 12:** The number of locations of EEG tensor components not correlated with musical feature.

	Prefrontal lobe	Temporal lobe	Parietal lobe	After the occipital lobe	Total
Normal group	97	24	3	21	145
Microconscious state group	44	70	51	37	202
Plant state group	51	118	86	52	307

RETRACTED

## Data Availability

The experimental data of this research are available from the author upon request.
